RETRACTED

# Sheltering of deleterious mutations explains the stepwise extension of recombination suppression on sex chromosomes and other supergenes

**DOI:** 10.1371/journal.pbio.3001698

**Published:** 2022-07-19

**Authors:** Paul Jay, Emilie Tezenas, Amandine Véber, Tatiana Giraud

**Affiliations:** 1 Université Paris-Saclay, CNRS, AgroParisTech, Ecologie Systématique et Evolution, 91190, Gif-sur-Yvette, France; 2 Univ. Lille, CNRS, UMR 8198 –Evo-Eco-Paleo, F-59000 Lille, France; 3 Université Paris Cité, CNRS, MAP 5, F-75006 Paris, France; University of Bath, UNITED KINGDOM

## Abstract

Many organisms have sex chromosomes with large nonrecombining regions that have expanded stepwise, generating “evolutionary strata” of differentiation. The reasons for this remain poorly understood, but the principal hypotheses proposed to date are based on antagonistic selection due to differences between sexes. However, it has proved difficult to obtain empirical evidence of a role for sexually antagonistic selection in extending recombination suppression, and antagonistic selection has been shown to be unlikely to account for the evolutionary strata observed on fungal mating-type chromosomes. We show here, by mathematical modeling and stochastic simulation, that recombination suppression on sex chromosomes and around supergenes can expand under a wide range of parameter values simply because it shelters recessive deleterious mutations, which are ubiquitous in genomes. Permanently heterozygous alleles, such as the male-determining allele in XY systems, protect linked chromosomal inversions against the expression of their recessive mutation load, leading to the successive accumulation of inversions around these alleles without antagonistic selection. Similar results were obtained with models assuming recombination-suppressing mechanisms other than chromosomal inversions and for supergenes other than sex chromosomes, including those without XY-like asymmetry, such as fungal mating-type chromosomes. However, inversions capturing a permanently heterozygous allele were found to be less likely to spread when the mutation load segregating in populations was lower (e.g., under large effective population sizes or low mutation rates). This may explain why sex chromosomes remain homomorphic in some organisms but are highly divergent in others. Here, we model a simple and testable hypothesis explaining the stepwise extensions of recombination suppression on sex chromosomes, mating-type chromosomes, and supergenes in general.

## Abstract 2

Many organisms have sex chromosomes with large non-recombining regions that have expanded stepwise, but the reasons for this remain poorly understood. This study shows that a theoretical model based on the sheltering of recessive deleterious mutations by permanently heterozygous alleles can explain the formation and extension of non-recombining regions in sex chromosomes and supergenes.

RETRACTED

## Introduction

Sex chromosomes, mating-type chromosomes, and supergenes in general are widespread in nature and control striking polymorphisms, such as sexual dimorphism or color polymorphism, in many organisms, including humans [1–5]. Supergenes display puzzling genomic architectures, defined by extensive regions lacking recombination, encompassing multiple genes [3,4]. Sex chromosomes, in particular, often appear to have evolved by stepwise extension of nonrecombining regions, generating “evolutionary strata” of differentiation between haplotypes [4,6,7]. It is generally thought that the reason for this gradual expansion of recombination suppression on sex chromosomes is that selection favors the linkage of sex-determining genes to sexually antagonistic loci, i.e., with alleles advantageous in one sex but disadvantageous in the other [7–9]. However, theoretical concerns have been raised about this idea [10], and it has proved difficult to obtain empirical support for a role of antagonistic selection in the extension of recombination suppression [6,11,12]. Furthermore, a gradual expansion of recombination suppression has been observed around many fungal mating-type loci [5] and at other supergenes, such as those controlling wing color in butterflies or social structure in ants [13,14]. Some type of antagonistic selection may exist between morphs determined by color or social supergenes, but antagonistic selection between fungal mating types is highly unlikely, given their life cycles and the results of genomic investigations [15,16]. For example, there has been repeated stepwise extensions of recombination suppression in anther-smut fungi despite the lack of a haploid phase consisting of cells of different mating types potentially expressing contrasted life history traits, leaving little room for antagonistic selection [15,16]. Alternative explanations have been put forward for the expansion of nonrecombining regions on sex chromosomes [11], such as meiotic drive [17], genetic drift [18], deleterious-mutation sheltering [19,20], and the neutral accumulation of sequence divergence [21], but the conditions in which such mechanisms could apply also appear to be restricted.

We develop here a general model for testing the idea that recombination suppression may extend stepwise around sex-determining or mating-type loci because it provides the fitness advantage of sheltering deleterious mutations segregating in nearby regions. Related hypotheses have been explored before, but in the restricted specific context of inbreeding [19,20]. We model here a more general hypothesis, based on the idea that genomes carry numerous deleterious recessive variants, as suggested by studies in a wide range of biological systems and by the pervasiveness of inbreeding depression in nature [22–27]. We use mathematical modeling and stochastic simulations to test the hypothesis that permanently heterozygous alleles, such as male-determining alleles in XY systems, protect linked chromosomal inversions against the expression of their recessive mutation load, potentially leading to an accumulation of inversions around permanently heterozygous alleles, generating evolutionary strata.

RETRACTED

The rationale behind this model is illustrated in Fig 1. Consider a diploid population carrying partially recessive, deleterious mutations. The combined effects of recombination, mutation, selection, and drift result in individuals carrying different numbers of deleterious variants genome-wide and within particular genomic regions (Fig 1A). Chromosomal inversions may occur at any position and suppress recombination when heterozygous, thereby capturing a specific combination of deleterious variants (i.e., a haplotype). Inversions capturing fewer deleterious variants than the population average for the region concerned have a fitness advantage and should, therefore, increase in frequency. Such inversions are advantageous due to associative overdominance, i.e., the inversion itself is neutral but it captures a combination of alleles that is advantageous when heterozygous [28,29]. However, as the frequency of an inversion increases, homozygotes for this inversion become more common. Homozygotes are at a strong disadvantage due to the recessive deleterious variants carried by these inversions, and selection against homozygotes would therefore be expected to prevent such inversions from reaching high frequencies (Fig 1B).

**Fig 1:** Schematic diagram of the model. (**A**) Within any population and for any genomic region, diploid individuals (here represented by 2 homologous chromosomes) and haplotypes (i.e., combinations of mutations, here one chromosome) carry variable numbers of partially recessive, deleterious mutations. A substantial fraction (about 50%) of haplotypes have fewer deleterious mutations than the average and should be favored by selection. Chromosomal inversions therefore have a significant chance of capturing beneficial haplotypes. (**B**) The increase in frequency of a beneficial inversion leads to an increase in the frequency of homozygotes for the inversion, which have a fitness disadvantage because they are homozygous for all the deleterious recessive mutations carried by the inversion. The fitness of the inversion therefore decreases with increasing inversion frequency, keeping the frequency of the inversion low. (**C**) Permanent heterozygosity at a Y-chromosome sex-determining allele protects linked inversions from this disadvantage of homozygosity. Hence, beneficial inversions (carrying fewer deleterious mutations than average) should spread and become fixed in the population of Y chromosomes. (**D**) Unlike those on autosomes, inversions capturing the Y sex-determining allele never suffer from homozygous disadvantage and should therefore accumulate on proto-Y chromosomes, leading to a suppression of recombination between the X and Y chromosomes. A similar mechanism should operate for any recombination suppressor acting in *cis* (not just chromosomal inversions) and any locus with permanently heterozygous alleles.

RETRACTED

Now, consider an inversion that, by chance, captures a permanently heterozygous allele, such as the male-determining allele in an XY system. If this Y-linked inversion captures fewer deleterious variants than the population average, it should increase in frequency without ever suffering the deleterious consequences of having its load expressed. The recessive deleterious mutations captured by the sex-linked inversion are, indeed, fully associated with the permanently heterozygous, male-determining allele, and will, therefore, never occur as homozygotes. Unlike autosomal inversions, Y-linked inversions retain their fitness advantage with increasing frequency (Fig 1C). Hence, Y-linked inversions with a lower load than average would be expected to spread, becoming fixed in the population of Y chromosomes, resulting in a suppression of recombination between the X and Y chromosomes in the region covered by the inversion.

The successive fixation of additional inversions linked to this Y-fixed inversion should cause the nonrecombining region to expand further, by the same process, thereby leading to the formation of a chromosome with a large nonrecombining region around the sex-determining locus—i.e., a sex chromosome with evolutionary strata of differentiation (Fig 1D). We use the term “chromosomal inversions” here for simplicity, but the proposed mechanism would hold for any mechanism suppressing recombination, and we model several types of recombination suppressors. The proposed mechanism would be expected to apply to any genomic region with a permanently or near-permanently heterozygous allele, such as mating-type loci in fungi or supergenes in many organisms. The accumulation of deleterious mutations following recombination suppression has been extensively studied [30–33], but we investigate here its converse: that deleterious mutations could be a cause, and not only a consequence, of recombination suppression. We also investigate whether this mechanism of deleterious mutation sheltering can explain the fusions sometimes observed between sex chromosomes and autosomes [20,34–36] and we explore the impact of various parameters on the probability of recombination suppression.

RETRACTED

## Results

We explored this general hypothesis of stepwise recombination suppression around permanently heterozygous alleles with infinite population deterministic models and individual-based simulations. Very little is known about the dynamics of deleterious mutations in genomic regions under particular recombination regimes, such as those generated by polymorphic inversions. We therefore had to use simulations to explore realistic scenarios involving various levels of drift. In both the infinite population model and individual-based simulations, we modeled diploid populations with only partially recessive deleterious mutations, occurring at a rate *u*, with heterozygous and homozygous individuals suffering from *1-hs* and *1-s* reductions in fitness, respectively, and with multiplicative effects of mutations on fitness. We first considered that all mutations occurring in genomes had the same dominance (*h*) and selection (*s*) coefficients, and then relaxed this hypothesis. Individuals were considered to have 2 pairs of chromosomes, one of which harbored a locus with at least 1 allele permanently or almost permanently heterozygous (see Methods for details). Several situations were considered, mimicking those encountered in XY sex-determination systems, in fungal mating-type systems and in overdominant supergenes. We analyzed the evolution of recombination modifiers suppressing recombination across the fragment in which they reside (i.e., *cis-*modifiers), either exclusively in heterozygotes (mimicking for example chromosomal inversions), or in both heterozygotes and homozygotes (e.g., histone modifications). Each of these recombination modifiers, which was assumed to be neutral in itself, appeared in a single haplotype, and was, thus, in linkage disequilibrium with a specific set of mutations, such that its fitness was exclusively dependent on the number of deleterious alleles within the segment captured. We first compared the dynamics of inversion-mimicking mutations in an autosome with those capturing a male-determining allele in an XY system (males are XY and females are XX, the male-determining allele being permanently heterozygous), and we then considered other types of recombination modifiers and heterozygosity rules.

RETRACTED

### Inversions less loaded than average are frequent in genomes

As noted by several authors [28,37,38], inversions capturing fewer deleterious mutations than the population average should increase in frequency. In infinite populations, the number of mutations harbored by individuals within a genomic segment with *n* sites follows a binomial distribution of parameters *n* and *q*, with *q* the mean frequency of mutations at mutation-selection equilibrium (Figs 2A and S1). On average, individuals harbor *nq* mutations on each of their chromosomal segments of size *n*. Under realistic parameter values, the vast majority of large chromosomal regions therefore carry several deleterious mutations. For example, considering *s* = 0.001, *h* = 0.1, *μ* = 10^−9^, and *n* = 2 Mb, more than 99.999% of chromosomal fragments carry a least 1 mutation, the mean number of mutations being *nq* = 20 (S1 Fig). If *m* is the number of recessive deleterious mutations captured by a given inversion, the mean fitness of individuals homozygous for the inversion (*W*_*II*_), heterozygous for the inversion (*W*_*NI*_), or lacking the inversion (*W*_*NN*_) in an infinite population can be easily expressed as a function of *n*, *q*, *h*, *s*, and *m* (see Methods; [28,37]). Once formed, inversions should increase in frequency if heterozygotes for the inversion are fitter than homozygotes without the inversion (*W*_*NI*_>*W*_*NN*_), which is the case if the inversion carries fewer mutations than the population average [*m*<*nq;* [28]].

**Fig 2:** In infinite populations, all less-loaded chromosomal inversions become fixed on the Y sex chromosome, whereas most remain at a low frequency on the autosome. (**a**) Expected number of segregating recessive deleterious mutations within a segment of *n* = 2 Mb as a function of the dominance coefficient (*h*), selection coefficient (*s*), and mutation rate (*u*). Mutations were considered to be at mutation-selection equilibrium frequency (see Methods). Parameters resulting in 1 and 2 expected mutations are highlighted by red and white lines, respectively, and are also shown on panels b and d. (**b**) Probability of occurrence of a less-loaded inversion covering a segment of *n* = 2 Mb as a function of the dominance coefficient (*h*), selection coefficient (*s*), and mutation rate (*u*). Less-loaded inversions are defined as those for which *m*<*nq*, where *m* is the number of mutations in the inversion (i.e., fewer than the average for the population). The number of mutations in inversions can take only integer values (*m* = 0, 1, 2, etc.), and the transition between these values affects the probability of occurrence of less-loaded inversions, yielding the noncontinuous graphs in panels b and d. (**c**) Deterministic change in inversion frequency, for the case of 2-Mb inversions capturing the male-determining allele on the Y-chromosome or inversions on an autosome. For clarity, the frequency displayed for Y-linked inversions is the frequency of inversions in the population of Y chromosomes. The figure illustrates the case of inversions carrying a number of mutations 5% lower than the population average (*m* = 0.95×*nq*), mutations being at their mutation-selection equilibrium frequency with *μ* = 10^−8^ and *h* = 0.1. S4 to S8 Figs illustrate the fate of inversions with intermediate degrees of linkage to the male-determining allele, with various numbers of mutations relative to the population average, or inversions linked to a locus with variable heterozygosity rules or in the X chromosome population. (**d**) Expected equilibrium frequency of less-loaded 2-Mb inversions (i.e., with *m* = 0,1, 2, …, *nq*) capturing the male-determining allele, or on an autosome, weighted by their probability of occurrence (Methods, Eqs 5, 6 and 7). This panel extends the result from panel c for a range of dominance coefficients (*h*), selection coefficients (*s*), and mutation rates (*u*). As above, the frequency displayed for Y-linked inversions is the frequency of inversions on the population of Y chromosomes. Above the line *nq* = 1, the mean number of segregating mutations in a given inversion (of length *n*) is less than 1, indicating that all less-loaded inversions are mutation-free. Such inversions can also become fixed on autosomes, leading to an expected equilibrium frequency of 1 for both autosomes and the Y chromosome. S9 Fig shows the overall frequencies of all inversions, whether less or more loaded than average, and over a larger range of parameters. The scripts used to produce this figure are available on GitHub.

RETRACTED

Repeated sampling from binomial distributions with a wide range of parameters showed that more than half the inversions occurring in genomes captured fewer deleterious mutations than the population average (Fig 2B; hereafter referred to as “less-loaded inversions”). Indeed, the distribution of mutation number across individuals is almost symmetric when *nq* is high (as the binomial distribution converges to a normal distribution; e.g., S1 Fig), but, when *nq* is low, the distribution is zero inflated, increasing the probability of inversions being less loaded. Therefore, a substantial fraction of inversions occurring in genomes are beneficial when they form (i.e., when rare enough not to occur as homozygotes). For example, with *h* values ranging from 0 to 0.5 and *s* values ranging from 0.001 to 0.25, between 36% and 98% (mean = 70%) of the 2-Mb inversions occurring in the genome are beneficial, carrying fewer recessive deleterious mutations than average (Fig 2B). Simulations in finite populations of different sizes confirmed that most inversions (mean = 66% in the range of parameter values studied) had a fitness advantage upon formation. The simulations also showed that inversions could be favored if they captured mutations that were rarer than average (S2 and S3 Figs).

### Less-loaded inversions are much more likely to fix when they capture a Y-like male determining locus

The deterministic increase in frequency of an inversion (I) on an autosome or capturing an XY-like sex-determining locus can easily be determined with a 2-locus 2-allele model. For example, the change in frequency of an inversion on the proto-Y chromosome can be expressed as:

$$\Delta F_{YI}=\frac{F_{YI}(F_{XIf}W_{II}+(1-F_{XIf})W_{NI}-\bar{W_{m}})\pm rW_{NI}D}{\bar{W_{m}}},$$

where *F*_*XIf*_ is the frequency of the inversion on the proto-X chromosome in females, *r* is the rate of recombination between the inversion and the sex-determining locus, *D* is their linkage disequilibrium, and $\bar{W_{m}}$ is mean male fitness (Fig 2C; see Methods and S1 Appendix for details). Based on this model, and initially assuming that inverted and noninverted segments no longer accumulate deleterious mutations after their formation, i.e., *W*_*II*_, *W*_*NI*_, and *W*_*NN*_ are fixed parameters (this strong assumption is relaxed latter), we simulated the evolutionary trajectory of inversions on autosomes and of inversions capturing the male-determining allele on the Y chromosome under a wide range of parameter values. We found that the frequency of less-loaded inversions tended to remain low in autosomes, whereas these inversions became fixed in the population of Y chromosomes (Fig 2C), as expected according to our hypothesis.

We therefore expressed the equilibrium frequency of inversions (*F*_*equ*,*m*_, Fig 2D) as a function of *m*, the number of deleterious mutations carried by the inversion, to calculate the threshold values at which autosomal and Y-linked inversions could be maintained or fixed (see S1 Appendix). Assuming that *q*≪1 and *s*≪1, we found that inversions on autosomes become fixed when *m*<*qhn*/(1−*h*) whereas they should stabilize at a frequency of (*W_NI_* – *W_NN_*)/(2*W_NI_* – *W_NN_* – *W_II_*), the equilibrium frequency of an overdominant locus, when *qhn*/(1−*h*)<*m*<*nq* (see Methods). Inversions on autosomes capturing more than *qhn*/(1−*h*) recessive deleterious mutations do, indeed, suffer from a homozygote disadvantage (*W*_*NI*_>*W*_*II*_, S1 Fig), preventing them from reaching high frequencies (Fig 2C). This is the case for most autosomal inversions under realistic parameter values (e.g., *m*>*qhn*/(1−*h*) for more than 99.99% of inversions when *n* = 2 Mb, *μ* = 10^−9^, *h* = 0.1, and *s* = 0.001, S1 Fig). By contrast, permanently heterozygous alleles protect inversions from this homozygote disadvantage, allowing these inversions to become fixed. All inversions capturing the male-determining allele become, therefore, fixed if they carry fewer than average mutations (i.e., *m*<*nq*). Thus, contrary to the argument proposed in a previous study that only mutation-free inversions can become fixed [35], we found that inversions can carry deleterious mutations and nevertheless become fixed in the population, provided that they carry fewer than *qhn*/(1−*h*) mutations if they are located on autosomes and fewer than *nq* mutations if they capture a permanently heterozygous allele (on the Y chromosome, for example).

RETRACTED

The expected equilibrium frequency of all inversions occurring in a given genomic region can be expressed as:

$$[F_{equ}]=\sum_{m=0}^{n}P_{m}\times F_{equ,m}$$

with *P*_*m*_ being the probability of occurrence of inversions with *m* mutations and *F*_*equ*,*m*_ the equilibrium frequency of inversions with *m* mutations (Fig 2D; see Methods). For permanently heterozygous inversions, we, thus, have:

$$[F_{equ}]=\sum_{m=0}^{\left\lfloor nq\right\rfloor }(\begin{array}{c} n\\ m \end{array})q^{m}{\left(1-q\right)}^{n-m},$$

and for autosomal inversions:

$$[F_{equ}]=\sum_{m=0}^{\left\lfloor nq\frac{h}{1-h}\right\rfloor }(\begin{array}{c} n\\ m \end{array})q^{m}{\left(1-q\right)}^{n-m}+\sum_{m=\lfloor nq\frac{h}{1-h}\rfloor +1}^{\left\lfloor nq\right\rfloor }(\begin{array}{c} n\\ m \end{array})q^{m}{\left(1-q\right)}^{n-m}\frac{W_{NI}-W_{NN}}{2W_{NI}-W_{NN}-W_{II}}.$$

With a realistic range of parameters, inversions are much more likely to become fixed if they capture the male-determining allele on the Y chromosome than if they are unlinked to this allele (e.g., on an autosome; Figs 2C and 2D and S4 to S9). For example, with *μ* = 10^−9^, *h* = 0.1, *s* = 0.001, and *n* = 2 Mb, 47% of inversions occurring on the Y chromosome would be expected to become fixed, versus only 0.000045% of inversions on autosomes.

### Drift and mutation accumulation do not prevent Y-linked inversion fixation

If deleterious mutations continue to arise after the formation of the inversion, the dynamics of the inversion become harder to predict deterministically. In infinite populations, the accumulation of mutations after the formation of the inversion can be approximated by $P_{t}=\frac{\mu }{sh}+(P_{0}-\frac{\mu }{sh})e^{-sht}$, where *P*_*t*_ is the number of mutations in the inversion at time *t* ([28,37]; see also [39]). This assumes that inverted segments evolve under mutation-selection dynamics with recombination. However, such assumptions do not hold in many situations, in contrast to what has been assumed in a previous study [39]. Indeed, low-frequency inversions in finite populations should almost never occur as homozygotes and should therefore evolve with almost no recombination. This is also true for inversions capturing a permanently heterozygous allele, which never undergoes recombination. We confirmed by simulations that the above approximation for an infinite population strongly departs from the situation observed in finite populations (e.g., S13 Fig). In finite populations, low-frequency or permanently heterozygous inversions tend to evolve under a Muller’s ratchet-like dynamic, with the mean fitness of inversions decreasing in a stepwise manner due to the sequential loss, by drift, of the inverted haplotypes with the lowest mutational load. Following their formation, autosomal and Y-linked inversions tend to accumulate more mutations than the population average, contrasting with predictions for infinite populations (S13 Fig). Only inverted segments reaching relatively high frequencies in autosomes eventually recombine when homozygous, and their dynamics of mutation accumulation therefore involve a mixture of a Muller’s ratchet-like regime (when rare, at the start of their spread) and a mutation-selection-drift regime with recombination (when they reach intermediate frequencies). Little is known about the transition between these regimes [40,41]. We therefore used individual-based simulations to study the fate of inversions accumulating deleterious mutations. This also made it possible to relax the previous assumption [38] that the time to inversion fixation is much shorter than the time taken for the inversions to accumulate deleterious mutations. Individual-based simulations also made it possible to relax the assumption that all genomic positions are independent.

RETRACTED

Simulations of the spread of inversions in finite populations with recurrent mutation confirmed the tendency identified in the deterministic model without mutation accumulation: Over most of the parameter space, inversions are much more likely to spread if they capture the sex-determining allele on the Y chromosome than if they are located on autosomes (Figs 3 and S10 to S16). Many autosomal inversions carrying a mutation load segregated for hundreds of generations. For example, with *N* = 1,000, *s* = 0.01, *h* = 0.1, and *μ* = 10^−8^, 73 of 10,000 inversions of 2 Mb in length continued to segregate after 500 generations. However, all these autosomal inversions were lost at the end of the simulations (i.e., after 10,000 generations, Fig 3A). These inversions initially spread because, by chance, they had a lower-than-average mutation load, but their homozygote disadvantage prevented them from reaching fixation. They were eventually lost because they accumulated further mutations relative to noninverted segments (Figs 3B and S13).

By contrast, substantial fractions of less-loaded inversions capturing the permanently heterozygous sex-determining allele on the Y chromosome spread until they became fixed in the Y chromosome population; this was the case even for inversions that were not mutation-free (Figs 3 and S10 to S16). For example, for *s* = 0.01, *h* = 0.1, *μ* = 10^−8^, and *N* = 1,000, 49 of the 10,000 Y-linked inversions (2 Mb) became fixed in the Y chromosome population, whereas all inversions on the autosome were lost. New mutations occurred on Y-linked inversions, but they did not accumulate rapidly enough to prevent these 49 inversions from spreading and reaching fixation (Figs 3A and 3B and S13). Permanent heterozygosity effectively results in directional selection for the less-loaded inversions, and not only for those free from mutations (Fig 3), leading to rapid fixation before the accumulation of too many new deleterious mutations.

**Fig 3:** In finite populations, a substantial fraction of less-loaded chromosomal inversions on the Y sex chromosome become fixed, whereas all less-loaded inversion on autosomes are lost. (**a**) Change in inversion frequency in stochastic simulations of 1,000 individuals experiencing recessive deleterious mutations at a rate *μ* = 10^−8^, all mutations having the same dominance and selection coefficients (here, *h* = 0.1 and *s* = 0.01). The figure displays the frequency of 10,000 independent inversions on each of an autosome and a proto-Y chromosome, with each line representing a specific inversion (i.e., a simulation). The evolutionary trajectories of inversions of different sizes, in larger populations, on the X-chromosome or with other parameter combinations, are displayed in S10–S14 Figs. (**b**) Change in the mean number of mutations carried by the inverted segments in each of the 10,000 simulations. Each line represents 1 simulation. A zoom-view of the autosomal inversion dynamics is shown in S13 Fig. (**c**) Proportions, in stochastic simulations, of 2-Mb inversions that were fixed after 10,000 generations for different parameter value combinations. This extends the result from panel a to other values of dominance coefficient (*h*), selection coefficient (*s*), and mutation rate (*u*). For each parameter combination, we simulated 10,000 inversions of 2 Mb capturing a random genomic fragment. Only inversions not lost after 20 generations are considered here. Note that Y axes have different scales. Results for inversions of different sizes are shown in S15 Fig and results for different population sizes are shown in S16 Fig. The datasets and scripts used to produce this figure are available on Figshare (doi: 10.6084/m9.figshare.19961033) and GitHub.

RETRACTED

### Other systems with permanently heterozygous alleles, other recombination modifiers, and sex chromosome–autosome fusion

Similar results were obtained when: (i) 2 or more permanently heterozygous alleles segregated at a mating incompatibility locus, modeling plant self-incompatibility or fungal mating-type systems (S5 and S14 Figs; [5,42]); (ii) the alleles were not permanently heterozygous, but were strongly overdominant, thus occurring mostly in the heterozygous state, as for several supergenes controlling color polymorphism (S8 Fig; [13,43,44]); (iii) the fitness effects of mutations occurring across the genome were drawn from a gamma distribution (i.e., the mutations segregating in populations had different fitness effects; S17 Fig); (iv) recombination modifiers suppressed recombination even when homozygous, as for histone modifications or methylation [45], rather than solely when heterozygous, as for inversions (S14 Fig); and (v) the inversion was in strong but incomplete linkage with the permanently heterozygous allele (e.g., 0.1 cM away from the allele, S4 to S8 Figs). Our model can thus account for the existence of inversions very close, but not fully linked to a mating-type locus, as reported in the chestnut blast fungus [46,47].

In addition, we found that the sheltering of deleterious recessive mutations could also lead to the fusion of the permanently heterozygous sex chromosome with an autosome when the fusion was associated with an extension of the nonrecombining region to the newly fused autosome (S18 Fig).

### Population parameters impacting the probability of inversion spread and fixation: population size, mutation rate, recessiveness, cost of heterozygous inversion, and life cycle

As shown above, we found that neutral recombination modifiers spread in a very large range of conditions if they captured permanently heterozygous alleles (Figs 3C, S15 and S16). As expected, inversions were more easily fixed on the Y chromosome when the deleterious mutations segregating in the genome were more recessive (Figs 3C, S15 and S16). Furthermore, as for any variant, even beneficial inversions benefiting from a selective advantage could be lost by drift, the probability of such loss depending on population size and the relative fitness of the inversion, in terms of the number and type of mutations initially captured relative to the average for the population (Figs 3, S15 and S16). Inversions occurring in regions in which large numbers of mutations segregate are more likely than those in mutation-poor regions to capture many fewer mutations than average, and therefore to have a stronger relative advantage. In other words, inversions in mutation-dense regions have a wider fitness distribution. The probability of Y-linked inversion fixation thus increases with increasing inversion size, mutation recessiveness, and mutation rate (Figs 3C, S15, S16 and S19).

RETRACTED

As expected [48], we found that, with increasing population size, beneficial inversions took more generations to spread to fixation (S11 and S12 Figs). This longer time favored the further accumulation of deleterious mutations in inversions, lowering their fitness, and, in some cases, preventing their fixation. The probability of inversion fixation in the Y chromosome population was, therefore, inversely correlated with population size, but was always much higher than that of fixation on autosomes (S15 and S16 Figs).

Less-loaded inversions linked to a permanently heterozygous allele also spread when we assumed that inversion heterozygotes suffered from a fitness cost, for example, because of a decrease in fertility due to segregation issues during meiosis (S20 and S21 Figs). However, with a heterozygous cost, only inversions with much fewer mutations than average were beneficial and could spread, and not all less-loaded inversions (see Methods and S1 Appendix); large inversions were thus more likely to spread because, compared to small inversions, they were more likely to carry much fewer mutations than average (S20 and S21 Figs).

Less-loaded inversions linked to a permanently heterozygous allele could also spread and fix in simulations assuming a haplodiplontic life cycle (i.e., an alternation of haploid and diploid phases) (S22 and S23 Figs). However, the occurrence of a haploid phase enhanced the purge of deleterious recessive mutations, leading to a lower population mutation load and thereby to a narrower fitness distribution of inversions upon formation (S23 Fig; [49,50]). A lower proportion of inversions were therefore fixed in haplodiplontic populations than in purely diploid populations (S22 Fig).

### Evolution of nonrecombining sex chromosomes with evolutionary strata despite possible reversions

We have shown above that inversions are likely to fix when capturing a permanently heterozygous allele, which should lead to their accumulation around such alleles and, for example, to the formation of nonrecombining sex chromosomes with a typical pattern of evolutionary strata. We studied the formation of such strata by the sequential occurrence of multiple inversions by simulating the evolution of large chromosomes experiencing the occurrence of multiple chromosomal inversions that can overlap with each other, under parameter values typical of those observed in mammals (Figs 4, 5 and S24). We simulated, over 100,000 generations, populations of *N* = 10,000 or *N* = 1,000 individuals, carrying two 100-Mb chromosomes, one of which harbored a mammalian-type sex-determining locus (XY males and XX females). Individuals experienced only deleterious or weakly deleterious mutations, with mutation rates and fitness effects similar to those observed in humans (fitness effect being drawn from a gamma distribution). The dominance coefficient of each mutation was chosen uniformly at random from a wide set of values (see Methods for details). At the start of each simulation, we randomly sampled *k* genomic positions that could be used as inversion breakpoints, with *k* being 10, 100, 1,000, or 10,000. These genomic positions represent inversion hotspots, such as those that can be generated by repeats in genomes [51]. In each generation, we introduced *j* inversions, *j* being sampled from a Poisson distribution. Simulation times were limited by using inversion rates such that one inversion, on average, occurred in each generation, throughout the whole population. The 2 breakpoints of each inversion were chosen, at random, from the k positions. It was, therefore, possible for 2 independent inversions to appear at the same position, allowing, in particular, the reversion of an inversion to its ancestral orientation, thereby restoring recombination. Reversion may be favored if an inversion has accumulated enough deleterious mutations after its fixation on the Y chromosome to carry a larger number of mutations than the population average [52]. We assumed that inversions partially overlapped by another inversion or that captured a smaller inversion could not be reversed, i.e., recombination could not be restored in such situations even if subsequent inversions reused the same breakpoints. Indeed, reversions of partially overlapped inversions do not restore ancestral arrangements but instead result in complex reshufflings of gene order and orientation and are therefore unlikely to restore recombination. We ran 10 simulations for each set of parameters.

RETRACTED

In all simulations assuming relatively large numbers of potential inversion breakpoints (*k* = 100, 1,000, 10,000), the Y chromosome progressively stopped recombining with the X chromosome as it accumulated inversions fully linked to the male sex-determining allele (Figs 4, 5 and S24). After the occurrence of an initial inversion capturing the male sex-determining allele, multiple inversions partially overlapping this inversion or other Y-fixed inversions were selected, thereby generating a growing chaos of overlapping chromosomal rearrangements. The nonrecombining region, thus, extended around the sex-determining locus in a stepwise manner, perfectly reflecting the evolution of sex chromosomes and other supergenes with evolutionary strata (Fig 4). Some events in the gradual extension of recombination suppression were reversed, due to the occasional occurrence of beneficial reversions (Figs 4 and 5). The accumulation of overlapping inversions was, however, more rapid than the occurrence of beneficial reversions, leading to a progressive extension of the nonrecombining region (Figs 4 and 5). By contrast, when we assumed a smaller number of potential breakpoints (*k* = 10), recombination suppression between sex chromosomes evolved in only 2 of the 10 simulations, and across only a small genomic region (Fig 5), owing to the more frequent occurrence of beneficial reversions.

**Fig 4:** Successive accumulation of inversions around a male-determining allele in an XY system, leading to the formation of nonrecombining sex chromosomes. A simulation of *N* = 1,000 individuals, each with 2 pairs of 100-Mb chromosomes, over 100,000 generations. Chromosome 1 harbors an X/Y sex-determining locus at 50 Mb (individuals are XX or XY). In each generation, one inversion appears, on average, in the whole population, in a randomly sampled individual, with the 2 recombination breakpoints sampled uniformly at random from *k* = 100 potential breakpoints. (**a**) Overview of chromosomal inversion frequency and position for 10 different generations. The width of the box represents the position of the inversion, and the height of the box indicates inversion frequency. Inversions appearing on the Y chromosome are depicted in yellow, those appearing on the X chromosomes are depicted in gray. The colors are not entirely opaque, so that regions with overlapping inversions appear darker. Previously fixed inversions may be lost due to the occurrence of beneficial reversions and selection. (**b**) Changes in the relative rate of recombination over the entire course of the simulation. The numbers of recombination events occurring at each position (binned in 1-Mb windows) are recorded at the formation of each offspring, across all homologous chromosomes in the population. Only recombination events between the X and the Y chromosomes are shown for chromosome 1 (i.e., recombination events between the two X chromosomes in females are not shown). Unlike chromosome 1, chromosome 2 harbors no permanently heterozygous alleles. All inversions on this chromosome suffer from homozygote disadvantage and very few inversions therefore become fixed on chromosome 2. See S24 Fig for a simulation with *N* = 10,000 individuals. The datasets and scripts used to produce this figure are available on Figshare (doi: 10.6084/m9.figshare.19961033) and GitHub.

RETRACTED

**Fig 5:** Effect of the number of potential inversion breakpoints on the evolution of recombination suppression at sex chromosomes. For each number of breakpoints, 10 simulations were conducted. Each dot represents the result of a simulation with *N* = 1,000 individuals. See Fig 4 for an example of such a simulation. (**a**) Fraction of the length of the Y sex chromosome not recombining after 100,000 generations. (**b**) Number of reversions occurring over the course of the 100,000 generations. Boxplot elements: central line: median, box limits: 25th and 75th percentiles, whiskers: 1.5× interquartile range. The dataset and script used to produce this figure are available on Figshare (doi: 10.6084/m9.figshare.19961033) and GitHub.

## Discussion

### Evolution of recombination suppression around permanently heterozygous alleles

Our results show that recombination suppression on sex chromosomes and other supergenes can evolve simply because genomes harbor many partially recessive, deleterious variants. Our model for the evolution of sex chromosomes, and supergenes in general, is based on simple and widespread phenomena: (i) inversions (or any recombination suppressor) can be favored solely because they contain fewer deleterious mutations than the population average, a situation applying to a substantial fraction of the inversions formed; (ii) such inversions tend to display overdominance: They are beneficial in the heterozygous state but suffer from a homozygote disadvantage, which prevents them from reaching high frequencies and becoming fixed on autosomes; and (iii) when, by chance, inversions capture a permanently heterozygous allele, they do not suffer from this homozygote disadvantage and are therefore able to spread until they are fully associated with the permanently heterozygous allele (e.g., they become fixed in the Y chromosome population). These 3 phenomena have been reported independently in several studies, but, to our knowledge, never in interaction (see references [28,38] for (i), [29,53] for (ii), and [5,19] for (iii)). The combined influence of the mechanisms related to (ii) and (iii) has been shown to promote sex chromosome–autosome fusion in highly inbred populations [20]. We show here that such mechanisms can readily lead to the stepwise extension of the nonrecombining region on sex chromosomes themselves, without the need for inbreeding. Moreover, unlike previous studies (e.g., [18,38,54]), we show that the higher probability of inversion fixation on Y chromosomes is not restricted to mutation-free inversions, but applies to any inversion capturing fewer deleterious mutations than the average. The proposed mechanism of deleterious mutation sheltering can also explain the fusions sometimes observed between sex chromosomes and autosomes, with the recombination suppression extending to a part of the fused autosome [20,34–36].

RETRACTED

The theory proposed here to explain the stepwise evolution of recombination suppression applies to any locus with at least 1 permanently or nearly permanently heterozygous allele. It only requires that, within a population, individuals carry different numbers of partially recessive deleterious mutations in a genomic region that can be subjected to recombination suppression. This situation is probably frequent in diploid, dikaryotic, or heterokaryotic organisms. For example, the mean distance between 2 heterozygous positions is approximately 1,000 bp in primates [55], and most mutations are likely partially recessive and deleterious [22,56]. Chromosomal rearrangements spanning hundreds of kilobases are frequently observed [51,57,58], and would, therefore, be expected to capture several deleterious variants.

### Mutation accumulation and inversion reversions are unlikely to prevent recombination suppression extensions

On autosomes, inversions maintained at low frequencies because of their homozygote disadvantage tend to be lost rapidly because they accumulate further deleterious mutations. On the Y chromosome, contrary to previous suggestions [28], we show that the accumulation of further deleterious mutations following the formation of an inversion is generally too slow to prevent the fixation of less-loaded inversions. Deleterious mutations nevertheless accumulate following fixation of the inversion, leading to Y-linked inversion degeneration, as observed on many nonrecombining sex chromosomes [30]. This may lead to selection for reversion of the inversion, thereby restoring recombination [52]. The question as to whether this can actually occur is common to all mechanisms explaining evolutionary strata, including sexual antagonism.

We found inversion reversion to be rare, unless there were no more than 10 inversion breakpoints over the two 100-Mb chromosomes. Indeed, for reversions to invade the population and restore recombination, the following conditions must be met: (i) sufficient deleterious mutations must accumulate in the initial inversion to render reversion beneficial; and (ii) a partially overlapping inversion should not have invaded the population before the occurrence of a beneficial reversion. Indeed, partially overlapping inversions result in a complex reshuffling of gene order and orientation, preventing the restoration of recombination even in situations in which reversion could be selected. When the number of potential breakpoints is relatively high, the probability of partially overlapping inversions occurring is higher than the probability of a reversion occurring, regardless of the relative rates of inversions and deleterious mutations.

RETRACTED

The reversion of inversions has been reported only in rare cases in which inversions occur at specific breakpoints rich in repeated elements [59,60], as in our simulations when assuming only a few possible breakpoints in the genome. The number of genomic positions at which inversions can occur in natural conditions is unknown, but this number is likely to be high given the chaos of rearrangements observed in some sex and mating-type chromosomes with hundreds of different breakpoints [16,51,61,62]. A recent study reported not only the recurrent appearance of inversions at the same positions, but also the existence of numerous potential breakpoints of inversions in human genomes [51]. Moreover, chromosomal rearrangements rapidly accumulate in recently established regions of nonrecombination [61] and overlapping inversions are observed on many sex chromosomes, which should prevent the restoration of recombination by reversions [16,62–65]. Therefore, over a wide range of realistic parameter values, the reversion of inversions should not prevent the stepwise formation of nonrecombining sex chromosomes. When there are few potential inversion breakpoints in the genome, the mechanism stabilizing inversions through dosage compensation considered in a recent model [52] may act in addition to the mechanism of sex-chromosome evolution studied here, as these 2 mechanisms are not mutually exclusive. However, by contrast to the framework of our model, the dosage compensation mechanism requires a form of sexual antagonism arising from XY-like asymmetry (i.e., one sex being heterogametic and the other homogametic); this dosage compensation mechanism [52] cannot, therefore, explain evolutionary strata on fungal mating-type chromosomes or bryophyte UV sex chromosomes [5,62].

### Parameters restricting the extension of recombination suppression

Our model showed that recombination suppression could also evolve near supergenes carrying more than two permanently heterozygous alleles, such as plant self-incompatibility or mushroom (Agaricomycotina) mating-type loci. Such multi-allelic loci are however not known to often display extensions of recombination suppression beyond incompatibility loci [66]. This may be because the existence of multiple alleles allows the loss of degenerated alleles: If a permanently heterozygous allele evolves a large nonrecombining region, for example, because of an inversion fixation, and then degenerates through Muller’s ratchet-like processes, it can be lost by selection, in contrast to alleles in biallelic compatibility systems. In addition, recessive self-incompatibility alleles can be homozygous in sporophytic systems [67]. In multi-allelic systems, we therefore expect to observe extensions of recombination cessation only around permanently heterozygous alleles, i.e., dominant self-incompatibility alleles, and only rare, recent and nondegenerated inversions; long-read polymorphism sequencing data would allow testing this hypothesis.

RETRACTED

Assuming a reduced fertility in heterozygotes for the inversion due to segregation issues possibly arising during meiosis [68] decreased the probability of inversion fixation, as expected. We found that large inversions were more likely to spread and fix than small inversions as they were more likely to capture haplotypes with much fewer mutations than average, thereby compensating the heterozygous cost; larger inversions may however be also more likely to induce segregation issues, although little data is available to date.

Given the lack of knowledge about inversion rates in natural conditions and the computation challenge represented by the simulation of complex patterns of recombination, we used reasonably high inversion rates in our sex-chromosome evolution simulations, making it possible to observe the stepwise extension of a nonrecombining region within 100,000 generations. Recent studies suggested that inversions may not be too rare and that inversion breakpoints may be widely distributed throughout the genome [51,69–71]. The use of different inversion rates might result in much shorter or much longer times for the stepwise extension of the nonrecombining region, but should not change the final outcome. Of course, lower inversion rates and higher costs of inversions in terms of fertility in heterozygotes would lower the rate of inversion fixation. In nature, the stepwise extension of the nonrecombining region between sex or mating-type chromosomes often occurs over time scales of the order of tens of millions of generations (e.g., about 250 M years in human [50]), suggesting that the fixation of inversions may be relatively rare events.

RETRACTED

### Predictions regarding the variability of sex-chromosome structure across species

We show that inversions are more likely to spread in regions harboring many segregating deleterious mutations, in which they have a greater chance of capturing highly advantageous haplotypes. Our model therefore predicts that species harboring a large number of deleterious recessive variants, due to their small population size, short haploid phase, outcrossing mating system, high mutation rate, and mutation recessiveness, for example, will be more prone to the evolution of large nonrecombining regions with evolutionary strata on sex chromosomes than species with a low mutation load. In addition, in species with large population sizes, the time required for an inversion to become fixed may exceed the time for which the number of deleterious mutations in the inversion remains below average. This would prevent some inversions from becoming fixed, potentially lowering the rate of expansion of nonrecombining regions on sex chromosomes in species with large population sizes. Depending on mutation effects and on the relative rates of inversions and mutations, this could however be compensated by the occurrence of a higher number of inversions each generation in large populations. Variations in population size, mutation rate, length of haploid phase, and mating system (outcrossing versus selfing or inbreeding) across lineages may, therefore, account for the large number of different sex-chromosome structures in nature, with some organisms maintaining homomorphic sex chromosomes and others evolving highly differentiated sex chromosomes with multiple strata [1].

The more efficient purging of recessive deleterious mutations in species with an extended haploid phase [49,50] could therefore potentially account for the smaller nonrecombining regions observed on the sex chromosomes of plants and algae than in animals [72,73]. In fungi, evolutionary strata around mating-type genes have been reported mostly in species with biallelic mating systems and whose main life stage is dikaryotic, with a very brief or inexistent haploid stage [5]. So far, an extension of recombination suppression beyond the mating-type locus in a fungus with an extended haploid phase has only be reported in *Cryphonectria parasitica*, but dikaryotic individuals are also relatively frequently found in this species [46,74,75].

A test of our model could thus look for association between the size of nonrecombining regions or the number of evolutionary strata on sex chromosomes and estimates of the number of deleterious mutations segregating in genomes, or parameters predicting the accumulation of deleterious mutations, such as population size, mating systems, length of the haploid phase, and mutation rates.

RETRACTED

## Conclusions

Given its simplicity and wide scope of application, our model of sex chromosome evolution is a powerful alternative to other explanations [6], although the various theories are not mutually exclusive. The strength of our model lies in the absence of strong assumptions, such as sexually antagonistic selection, XY heterogamety asymmetry, or small population sizes. Our model, based on the often overlooked observation that recessive deleterious mutations are widespread in genomes within natural populations, can explain the evolution of stepwise recombination suppression over a wide range of realistic parameter values. Furthermore, it can explain why some supergenes, such as those in butterflies and ants, display evolutionary strata [13,14], and why many biallelic mating-type loci in dikaryotic fungi display a stepwise extension of nonrecombining regions despite the absence of sexually antagonistic selection or XY-like asymmetry in these organisms [5,16]. Our model can also explain why meiotic drivers, which are often permanently heterozygous, are often associated with large nonrecombining region involving polymorphic chromosomal inversions [76,77]. Our model therefore provides a general and simple framework for understanding the evolution of nonrecombining regions around many kinds of loci carrying permanently heterozygous alleles.

## Methods

### Infinite population deterministic model

We consider the discrete-time evolution of an infinite size, randomly mating population experiencing only deleterious recessive mutations, with heterozygotes and homozygotes suffering from a *1-hs* and *1-s* reduction in fitness, respectively. At all *n* sites, mutations are at the same mutation-selection equilibrium frequency, denoted by *q*. We used nonapproximated values of *q* as derived by [78]:

$$q=\frac{h(1+u)}{2(2h-1)}[1-\sqrt{1-\frac{4(2h-1)u}{sh^{2}{\left(1+u\right)}^{2}}}].$$

We assume that the sites are independent. The number of mutations carried by a chromosomal segment of length *n* then follows a binomial distribution of parameters (*n*, *q*). We follow the frequency of an inversion I of size *n*, considering that it captures *m* mutations and that it appears in a population carrying only noninverted segments. The mean fitness of a noninverted homozygote can be computed as follows (see S1 Appendix, section 2):

$$W_{NN}={\left(1-2q(1-q)hs-q^{2}s\right)}^{n}.$$

Note that in the parameter regimes where we can make the approximation *q*≈*u*/*hs* with *q*≪1, we have *W*_*NN*_≈(1−2*u*)^*n*^, in accordance with mutation load theory [37,79]. Similarly, an individual who is heterozygous for an inversion with *m* mutations has a mean fitness of:

$$W_{NI}={\left(q(1-s)+(1-q)(1-hs)\right)}^{m}{\left(q(1-hs)+1-q\right)}^{n-m}.$$

Assuming that *q*≪1, Nei and colleagues [28] considered that individuals heterozygous for an inversion had no homozygous mutations, so that $W_{NI}\approx {\left(1-hs\right)}^{m}{\left(1-hs\right)}^{nq}={\left(1-hs\right)}^{nq+m}$. Note that we use nonapproximated values in our computations. An individual who is homozygous for a segment I with *m* mutations is homozygous for all these mutations. Its fitness can therefore be expressed as:

$$W_{II}={\left(1-s\right)}^{m}.$$

The inversion frequency trajectory can be determined with a simple 2-locus 2-allele model. We considered 4 different situations, depending on the possible heterozygosity at the locus with permanently heterozygous alleles. The S1 Appendix, sections 4 to 8, presents the evolution in time of the frequency of the inversion in detail in these 4 situations. Here, we briefly describe the results for inversions more or less linked to a permanently heterozygous allele in a XY system. The change in frequency of inversions on the Y chromosome, on the X chromosome, or on autosomes between generations *t* and *t*+1 (Fig 2C) is described by

$$F_{XIm}^{t+1}=\frac{F_{XIf}^{t}(W_{II}F_{YI}^{t}+W_{NI}F_{YN}^{t})+rW_{NI}D^{t}}{\bar{W_{m}^{t}}},$$

$$F_{XNm}^{t+1}=\frac{F_{XNf}^{t}(W_{NN}F_{YN}^{t}+W_{NI}F_{YI}^{t})-rW_{NI}D^{t}}{\bar{W_{m}^{t}}},$$

$$F_{XIf}^{t+1}=\frac{F_{XIm}^{t}F_{XIf}^{t}W_{II}+\frac{1}{2}W_{NI}(F_{XIm}^{t}F_{XNf}^{t}+F_{XIf}^{t}F_{XNm}^{t})}{\bar{W_{f}^{t}}},$$

$$F_{XNf}^{t+1}=\frac{F_{XNm}^{t}F_{XNf}^{t}W_{NN}+\frac{1}{2}W_{NI}(F_{XNm}^{t}F_{XIf}^{t}+F_{XNf}^{t}F_{XIm}^{t})}{\bar{W_{f}^{t}}},$$

$$F_{YI}^{t+1}=\frac{F_{YI}^{t}(W_{II}F_{XIf}^{t}+W_{NI}F_{XNf}^{t})-rW_{NI}D^{t}}{\bar{W_{m}^{t}}},$$

$$F_{YN}^{t+1}=\frac{F_{YN}^{t}(W_{NN}F_{XNf}^{t}+W_{NI}F_{XIf}^{t})+rW_{NI}D^{t}}{\bar{W_{m}^{t}}},$$

$$F_{XI}=\frac{2}{3}F_{XIf}+\frac{1}{3}F_{XIm},$$

$$F_{I}=\frac{1}{4}F_{YI}+\frac{3}{4}F_{XI},$$ (Eq 1)

where $F_{YI}^{t}$ is the frequency of the inversion in the population of Y chromosomes at time *t*, $F_{XIf}^{t}$ is the frequency of the inversion on the X chromosome in females (respectively, $F_{XIm}^{t}$ in males), *r* is the rate of recombination between the inversion and the sex-determining locus, *D* is their linkage disequilibrium such that $D^{t}=F_{XNf}^{t}F_{YI}^{t}-F_{XIf}^{t}\;F_{YN}^{t}$, and $\bar{W_{m}^{t}}$ is the mean male fitness (Fig 2C; see S1 Appendix, section 8 for details). When *r* = 0.5, this system of equations describes the evolution of inversions on autosomes. Unless otherwise stated, the deterministic simulations presented here (Figs 2C and S4 to S8) were performed with an initial *D* = −0.01 or *D* = 0.01, depending on the allele which the inversion appeared linked to. Results for various initial linkage disequilibrium values are presented in S6 Fig. When the inversion captures the male-determining allele, *r* = 0, *F*_*XIm*_ = *F*_*XIf*_ = 0, and *F*_*XNf*_ = *F*_*XNm*_ = 1 at any time *t*. The equations for $F_{YI}^{t}$, the frequency of inversions capturing the male-determining allele then reduces to

$$F_{YI}^{t+1}=F_{YI}^{t}\frac{W_{NI}}{\bar{W_{m}^{t}}}$$

$$F_{YN}^{t+1}=F_{YN}^{t}\frac{W_{NN}}{\bar{W_{m}^{t}}}$$

with $\bar{W_{m}^{t}}=F_{YN}^{t}W_{NN}+F_{XI}^{t}W_{NI}$. Substituting *F*_*YN*_ by 1−*F*_*YI*_ and subtracting $F_{YI}^{t}$, we have $\Delta F_{YI}=\frac{F_{YI}^{t}(1-F_{YI}^{t})(W_{NI}-W_{NN})}{\bar{W_{m}^{t}}}$.

RETRACTED

The search for *F*_*YI*_ such that Δ*F*_*YI*_ = 0 readily gives 2 equilibria: 0 and 1. Since $\bar{W_{m}^{t}}>0$ and 0≤*F*_*YI*_≤1, we can conclude that:

If *W*_*NI*_>*W*_*NN*_, *F*_*YI*_→1,

if *W*_*NI*_<*W*_*NN*_, *F*_*YI*_→0.

In the case of an inversion appearing on an autosome (*r* = 0.5), *F*_*XIm*_ = *F*_*XIf*_ = *F*_*YI*_ and $\bar{W_{m}}=\bar{W_{f}}=\bar{W}$, so that the change in inversion frequency in the population is:

$$F_{I}^{t+1}=\frac{{\left(F_{I}^{t}\right)}^{2}W_{II}+F_{I}^{t}F_{N}^{t}W_{NI}}{\bar{W_{t}}}$$

and

$$\Delta F_{I}=\frac{F_{I}}{\bar{W}}(F_{I}^{2}(2\;W_{NI}-W_{II}-W_{NN})+F_{I}(W_{II}+2W_{NN}-3W_{NI})+W_{NI}-W_{NN})=\frac{F_{I}}{\bar{W}}\times P(F_{I}),$$

with $P(X)=X^{2}(2\;W_{NI}-W_{II}-W_{NN})+X(W_{II}+2W_{NN}-3W_{NI})+W_{NI}-W_{NN}$.

The equilibria are 0 and the roots of the polynomial P, which are 1 and $\frac{W_{NI}-W_{NN}}{2W_{NI}-W_{II}-W_{NN}}$. We thus have:

If *W*_*NI*_>*W*_*NN*_ and *W*_*II*_>*W*_*NI*_, then *F*_*I*_→1,

If *W*_*NI*_>*W*_*NN*_ and *W*_*II*_<*W*_*NI*_, then $F_{I}\to \frac{W_{NI}-W_{NN}}{2W_{NI}-W_{II}-W_{NN}},$

If *W*_*NI*_<*W*_*NN*_, then *F_I_*→0.

Inversion equilibrium frequencies therefore depend, as expected, on the relative fitness of homozygotes and heterozygotes for the inversion and of the noninverted homozygotes. We thus derive the conditions for the inversion to be favored or disfavored as a function of the number of mutations captured by the inversion (*m*). A straightforward computation gives (see the S1 Appendix, section 9):

*W*_*II*_>*W*_*NI*_ if and only if *m*<*β*_1_(*q*, *h*, *s*)×*n*,

*W*_*NI*_>*W*_*NN*_ if and only if *m*<*β*_2_(*q*, *h*, *s*)×*n*, with

$$\beta_{1}(q,h,s)=\frac{\ln\left(q(1-hs)+1-q\right)}{ln(\frac{\left(1-s)(q(1-hs)+1-q\right)}{q(1-s)+(1-q)(1-hs)})}=\frac{ln(1-qhs)}{\ln\left(\frac{\left(1-s)(1-qhs\right)}{1-hs-qs(1-h)}\right)},$$ (Eq 2)

$$\;\beta_{2}(q,h,s)=\frac{\ln\left(\frac{1-2q(1-q)hs-q^{2}s}{q(1-hs)+1-q}\right)}{\ln\left(\frac{q(1-s)+(1-q)(1-hs)}{q(1-hs)+1-q}\right)}.$$ (Eq 3)

Assuming *q*≪1 and *s*≪1, these quantities can be approximated by $\beta_{1}\approx q\frac{h}{1-h}$ and *β*_2_≈*q* (the latter in accordance with a previous study [28]). When $\frac{qhn}{1-h}<m<nq$, inversions should thus go to fixation on Y chromosomes and stabilize at intermediate frequency on autosomes. When $m<\frac{qhn}{1-h}$, inversions should go to fixation on autosomes and on the Y chromosome. Observe that the closer *h* is to ½ (i.e., the scenario without dominance), the smaller the difference between the thresholds *β*_1_ and *β*_2_ is. When *h* = 0.5, *β*_1_ = *β*_2_, inversions should therefore go to fixation on autosome when they have fewer mutations than average, as they have then no homozygous disadvantage preventing their fixation. In contrast, when *h* is small, *β*_1_ is significantly smaller than *β*_2_, showing that the condition for heterozygotes to be favored over noninverted homozygotes (*W*_*NI*_>*W*_*NN*_) is much easier to meet than for inversion homozygotes to be favored over inversion heterozygotes (*W*_*II*_>*W*_*NI*_): inversions are therefore much likely to be maintained at intermediate frequencies on autosomes than to fix. See S1 Fig for a graphical representation of these results and the S1 Appendix, section 9, for derivation details.

RETRACTED

We can use these equilibrium frequencies as functions of *m* to compute the expected equilibrium frequency of inversions that can occur in the genome (*F*_*equ*_, Figs 2D and S9). To do so, we sum for all *m*∈{0,…,*n*} the equilibrium frequencies of inversions (*F*_*equ*,*m*_) weighted by their occurrence probability (*P*_*m*_). For inversions on the Y chromosome, we therefore have:

$$[F_{equ}]=\sum_{m=0}^{n}P_{m}\times F_{equ,m}=\sum_{m=0}^{n}\left(\begin{array}{c} n\\ m \end{array}\right)q^{m}{\left(1-q\right)}^{n-m}F_{equ,m}=\sum_{m=0}^{\left\lfloor nq\right\rfloor }(\begin{array}{c} n\\ m \end{array})q^{m}{\left(1-q\right)}^{n-m}.$$ (Eq 4)

For inversions on autosomes, we obtain, using the approximate values for *β*_1_ and *β*_2_ derived earlier in the case *q*≪1 and *s*≪1:

$$[F_{equ}]=\sum_{m=0}^{\left\lfloor nq\frac{h}{1-h}\right\rfloor }(\begin{array}{c} n\\ m \end{array})q^{m}{\left(1-q\right)}^{n-m}+\sum_{m=\lfloor nq\frac{h}{1-h}\rfloor +1}^{\left\lfloor nq\right\rfloor }(\begin{array}{c} n\\ m \end{array})q^{m}{\left(1-q\right)}^{n-m}\frac{W_{NI}-W_{NN}}{2W_{NI}-W_{NN}-W_{II}}.$$ (Eq 5)

The expected equilibrium frequency of less-loaded inversions (Fig 2D) is therefore the expected equilibrium frequency of all inversions divided by the probability of occurrence of less-loaded inversions:

$$[F_{equ}^{less\;loaded}]=\frac{\left[F_{equ}\right]}{\sum_{m=0}^{\left\lfloor nq\right\rfloor }P_{m}}=\frac{\left[F_{equ}\right]}{\sum_{m=0}^{\left\lfloor nq\right\rfloor }(\begin{array}{c} n\\ m \end{array})q^{m}{\left(1-q\right)}^{n-m}}.$$ (Eq 6)

The fate of inversions associated with a heterozygote fitness cost is described in section 10 of the S1 Appendix.

RETRACTED

### Individual-based simulations

We used SLiM V3.2 [80] to simulate the evolution of a single panmictic population of *N* = 1,000 or *N* = 10,000 individuals in a Wright–Fisher model. To assess the fate of inversions under various conditions (Fig 3), we simulated individuals with 2 pairs of 10-Mb chromosomes on which mutations occurred at a rate *u*, with *u* ranging from 10^−6^ to 10^−9^ per bp, their dominance coefficient *h* ranged from 0 to 0.5 (0, 0.01, 0.1, 0.2, 0.3, 0.4, 0.5) and their selection coefficient *s* from −0.5 to 0 (0, −0.001, −0.01, −0.1, −0.25, −0.5). The main and supplementary figures show the results for *μ* = 10^−8^ and *μ* = 10^−9^ unless otherwise stated. We also simulated populations where each occurring mutation had its selection coefficient *s* drawn from a gamma distribution with a shape of 0.2, and its dominance coefficient *h* randomly sampled among 0, 0.001, 0.01, 0.1, 0.25, 0.5 with uniform probabilities (S17 Fig). We considered recombination rates of 10^−6^ and 10^−5^ per bp, which gave similar results. Results are presented for analyses in which the recombination rate was 10^−6^. Among the 5,000,000 sites on chromosome 1, a single segregating locus was subject to balancing selection, for which several situations were considered: (i) the locus had 2 alleles, only one of which was permanently heterozygous, mimicking a classical XY (or ZW) determining system (Fig 3); (ii) the locus had 2 permanently heterozygous alleles, mimicking, for example, the situation encountered at most fungal mating-type loci; (iii) the locus had 3 (or more) permanently heterozygous alleles, mimicking, for example, the situation encountered in plant self-incompatibility systems and mushroom (Agaromycotina) mating-type loci.

For each parameter combination (*u*, *h*, *s*, *N*, heterozygosity rule at the locus with a permanently heterozygous allele), a simulation was run for 15,000 generations to allow the population to reach an equilibrium for the number of segregating mutations. S25 Fig shows that each population had reached equilibrium by the end of the burn-in period. The population state was saved at the end of this initialization phase. These saved states (one for each parameter combination) were repeatedly used as initial states for studying the dynamics of recombination modifiers. Recombination modifiers mimicking inversions of 500 kb, 1,000 kb, 2,000 kb, and 5,000 kb were then introduced on chromosome 1 around the locus under balancing selection (X-linked or Y-linked inversions) or on chromosome 2 (autosomal inversions). For each parameter combination (*h*, *s*, *u*, *N*, heterozygosity rule, size of the region affected by the recombination modification and position on the genome), we ran 10,000 independent simulations starting with the introduction of a single recombination modifier in the same saved initial population. These inversion-mimicking, recombination modifier mutations were introduced on a single, randomly selected chromosome and, when heterozygous, they suppressed recombination across the region in which they reside (i.e., as a *cis*-recombination modifier). We monitored the frequency of these inversion-mimicking mutations during 10,000 generations, during which all evolutionary processes (such as point mutation, recombination, and mating) remained unchanged, e.g., mutations were still appearing on inversions following their formation. Under the same assumptions and parameters, we also studied the dynamics of recombination modifiers suppressing recombination also when homozygous and not only when heterozygous, again across a fragment in which they reside (S14 Fig).

RETRACTED

To study the effect of the existence of a haploid phase on the accumulation of deleterious mutations and the spread of inversions on autosomes and sex chromosomes, we performed additional simulations, involving 15,000 generations of burn-in and the introduction of 10,000 inversions under each combination of parameters in these initial populations, as above. The populations were considered to harbor a single locus with 2 permanently heterozygous alleles (similarly to the previous situation (ii)). Every x generation, populations experimented a haploid generation, with x taking the values 2, 3, 5, 10, or 100. For simulating haploidy, all mutations from one chromosome of each pair (“genome2” in SLiM) were removed, and the dominance coefficient of mutations on the other chromosome (“genome1” of each pair) was set to 1. The recombination rate was set to 0, and mating could only occur between gametes that were derived from the first chromosome of each pair. Therefore, during haploid generations, selection acted only on the first chromosome of each pair, and the second chromosome had no contribution to the following generation. These modifications allowed simulating the occurrence of haploid phases without changing most parameters or model behavior. Note that, during the haploid phase, the number of individuals remained unchanged, but the number of haploid genomes was divided by 2, because the second haploid genome of each pair had no contribution to the following generation.

RETRACTED

To study the evolution of chromosomal fusion (S18 Fig), we simulated populations with no recombination between X and Y chromosomes (chromosome 1) between the position 1 Mb and 9 Mb during 15,000 generations (burn-in), mimicking the evolution of a population with old sex chromosomes and small pseudoautosomal regions (1 Mb on each chromosome edge). Then, we introduced a fusion-mimicking mutation resulting in the linkage of 1 sex chromosome (chromosome 1, X or Y) and 1 autosome (chromosome 2), and suppressing the recombination when heterozygous over 1 Mb of the fused side of each chromosome (see S18 Fig for a graphical representation). Therefore, these mutations behave like 2-Mb inversions that would also lead to chromosome fusion and result in the extension of the size of the nonrecombining region from 8 Mb to 10 Mb. We tracked the frequency of 10,000 X-autosome and Y-autosome fusion-mimicking mutations for each parameter combination (as done before for inversion-mimicking mutations).

To study more specifically the formation of evolutionary strata on sex chromosomes (Figs 4 and 5), we also simulated the evolution of two 100-Mb chromosomes, one of which carried an XY sex-determining locus at the 50-Mb position, over 115,000 generations (including an initial burn-in of 15,000 generations): individuals could be either XX or XY and could only mate with individuals of a different genotype at this locus. We simulated randomly mating populations of *N* = 1,000 and *N* = 10,000 individuals. Point mutations appeared at a rate of *μ* = 10^−9^ per bp, and their individual selection coefficients were determined by sampling a gamma distribution with a mean of −0.03 and with a shape of 0.2; these parameter values were set according to observations in humans [22,81]. For each new mutation, a dominance coefficient was chosen from the following values, considered to have uniform probabilities: 0, 0.001, 0.01, 0.1, 0.25, 0.5. At the beginning of each simulation, we randomly sampled *k* genomic positions over the 2 chromosomes that could be used as inversion breakpoints, with *k* being 10, 100, 1,000, or 10,000. After the 15,000 generations of the burn-in period allowing populations to reach an equilibrium in terms of the number of segregating mutations, we introduced each generation *j* inversions in the population, *j* being sampled from a Poisson distribution of parameter *λ*, with *λ* = *N*×*k*×*u*_*i*_, *u*_*i*_ being the inversion rate. In order to keep the simulation time tractable, we used inversion rates allowing 1 inversion to occur on average each generation in the population (i.e., *N*×*k*×*u*_*i*_ = 1). For each inversion, the first breakpoint was randomly chosen among the *k* positions, and the second among the potential breakpoint positions less than 20 Mb apart on the same chromosome (considering therefore only a subset of the *k* positions for the second breakpoints). Two independent inversions could use the same breakpoints, allowing in particular inversion reversion restoring recombination. If 2 independent inversions occurred with the same breakpoints on different haplotypes (for example, on the X and on the Y chromosome), we assumed that recombination was restored between these haplotypes, as a reversion would do. The occurrence of partially overlapping inversions (i.e., with different breakpoints) on different haplotypes did not restore recombination between these haplotypes. We assumed that inversions subsequently partially overlapped by another inversion or that captured a smaller inversion could not reverse, i.e., the restoration of recombination by further inversions, even if using the same breakpoints, was prevented. (For *N* = 1,000, for each values of *k* (i.e., 10, 100, 1,000, 10,000), we ran 10 simulations (Fig 5). For *N* = 10,000, because of computing limitation (each simulation taking about 3 weeks to run), we only ran 1 simulation per number of breakpoints.

RETRACTED

Simulations were parallelized with GNU Parallel [82].

## Supporting information

S1 Fig Distribution of the occurrence probability of inversions depending on the number of mutations they capture. This figure represents the binomial distribution of the number of mutations on a segment of *n* = 2,000,000 sites, with mutations occurring at a rate *μ* = 10^−8^ and having selective effect of *s* = 0.01 and *h* = 0.1. The filling color of the distribution represents the expected state of the inversions on autosomes based on Eqs 2 and 3 (Methods). The probability of occurrence of an inversion carrying fewer than *m* = *qhn*/(1−*h*) mutations, and therefore fixing on the autosome (dark blue filling), is so low that it is not visible on this plot. The script used to produce this figure is available on GitHub.
(PDF)

S2 Fig Fate of neutral chromosomal inversions on autosomes depending on the relative number of mutations they carry compared to population average and the relative frequency of these mutations. Each dot represents a 2-Mb inversion on an autosome. For each parameter combination, the fate (i.e., being lost or still segregating) of 10,000 inversions after 1,000 generations in stochastic simulations of a population of *N* = 1,000 individuals is displayed depending on the number of mutations they captured upon formation relative to the population average. Only inversions not linked to a permanently heterozygous allele were considered. Results for sex-linked inversions are displayed in S3 Fig. The Y axis represents the number of mutations captured by the inversions upon formation relative to the mean number of mutations within the same region in noninverted segments. Dot color represents the mean of the frequencies (in the entire population) of the mutations captured by inversions relative to the mean of the frequencies (in the entire population) of mutations in noninverted segments: A blue dot represents an inversion capturing mutations rarer than average, whereas a red dot represents an inversion capturing mutations more frequent than average. Boxplot elements: central line: median, box limits: 25th and 75th percentiles, whiskers: 1.5× interquartile range. The vast majority of inversions still segregating after 1,000 generations carried fewer or rarer mutations than the population average. The dataset and script used to produce this figure are available on Figshare (doi: 10.6084/m9.figshare.19961033) and GitHub.
(PDF)

S3 Fig Fate of neutral chromosomal inversions linked to a permanently heterozygous allele depending on the relative number of mutations they carry compared to population average and the relative frequency of these mutations. Similar to S2 Fig but with inversions linked to a permanently heterozygous allele (such as a Y sex-determining allele). For each parameter combination, the fate (i.e., being lost or still segregating) of 10,000 inversions after 1,000 generations in stochastic simulations is displayed depending on the number of mutations captured upon formation relative to the population average. Dot color represents the mean of the frequencies (in the entire population) of the mutations captured by inversions relative to the mean of the frequencies (in the entire population) of mutations in noninverted segments: A blue dot represents an inversion capturing mutations rarer than average, whereas a red dot represents an inversion capturing mutations more frequent than average. Boxplot elements: central line: median, box limits: 25th and 75th percentiles, whiskers: 1.5× interquartile range. The vast majority of inversions still segregating after 1,000 generations carried fewer or rarer mutations than the population average. The dataset and script used to produce this figure are available on Fig share (doi: 10.6084/m9.figshare.19961033) and GitHub.
(PDF)

S4 Fig Deterministic trajectories of inversion frequency when in linkage with the sex-determining allele on the Y chromosome or on the X chromosome. Similar to Fig 2C, but considering both X-linked and Y-linked inversions, and various recombination rates between the sex-determining locus and inversions. Trajectory of inversions is represented for different values of the selection and dominance coefficients of their mutations and the linkage of these inversions to an X or to a Y sex-determining allele. Mutation frequencies are at mutation-selection equilibrium (see Methods) with a mutation rate of *μ* = 10^−8^. Inversions of 2 Mb are introduced with an initial linkage disequilibrium of *D* = 0.01 or *D* = −0.01, depending on whether they appear linked to the male-determining allele on the Y chromosome or to the female-determining allele on the X chromosome. The figure illustrates the case of inversions carrying a number of mutations 20% lower than the population average (*m* = ⌊0.8×*nq*⌋), as frequently observed (S1–S3 Figs). (**a**) Inversions appearing in linkage with a sex-determining allele on the Y chromosome (permanently heterozygous). The frequency of the inversion in the population of Y chromosomes is followed during the first 10,000 generations. Linkage strength is indicated by line colors (distance in cM between inversions and the sex-determining allele). Inversions at 50 cM from the sex-determining locus behave like inversions on autosomes. There is a nearly perfect overlap between curves representing the 1, 5, and 50 cM linkage cases, so that only 50 cM curves are visible. (**b**) Inversions appearing in linkage with the sex-determining allele on the X chromosome. The frequency of the inversion in the population of X chromosomes is followed during the first 10,000 generations. Linkage strength is indicated by line colors (distance in cM between inversions and the sex-determining allele). See S1 Appendix, section 8, for modeling details. The script used to produce this figure is available on GitHub.
(PDF)

S5 Fig Deterministic trajectory of inversion frequency depending on their initial mutation load and their linkage to a locus with 2 permanently heterozygous alleles. Similar to Figs 2C and S4 but considering inversions in linkage to a locus with 2 permanently heterozygous alleles (and not only 1 as in the XY systems), and various mutation loads associated with the inversions upon formation. Trajectory of inversions in an infinite population depending on the selection coefficient of the segregating mutations, the dominance coefficient of these mutations, and the linkage of these inversions to a permanently heterozygous locus with 2 alleles. Mutations are at mutation-selection equilibrium frequencies (see Methods) with a mutation rate of *μ* = 10^−8^. Inversions of 2 Mb are introduced with an initial linkage disequilibrium of *D* = 0.01. Inversions are linked to only 1 of the 2 alleles at the permanently heterozygous locus, and so even fully linked inversions can increase up to a maximum frequency of 50%. Linkage strength is indicated by line colors (distance in cM between inversions and permanently heterozygous locus). Inversions at distances larger than 50 cM from the sex-determining locus behave like inversions on autosomes. The figure illustrates the case of inversions carrying varying numbers of mutations compared to the population average. (**a**) Case of inversions with 20% fewer mutations than the population average (*m* = ⌊0.8×*nq*⌋00). (**b**) Case of inversions with 10% fewer mutations than the population average (*m* = ⌊0.9×*nq*⌋). (**c**) Case of inversions with 1% fewer mutations than the population average (*m* = ⌊0.99×*nq*⌋). In all cases, there is a nearly perfect overlap between curves representing the 1, 5, and 50 cM linkage cases, so that only 50-cM curves are visible. Individual-based simulations of the same system are shown in S14 Fig. See S1 Appendix, section 6, for modeling details. The script used to produce this figure is available on GitHub.
(PDF)

S6 Fig Deterministic trajectory of inversion frequency depending on their linkage to a permanently heterozygous locus with 2 alleles (in centimorgan) and on their initial association (initial linkage disequilibrium). Trajectory of inversions in infinite populations as a function of the selection coefficient of the segregating mutations, their linkage to a permanently heterozygous locus with 2 alleles, and the initial level of linkage disequilibrium (D) between the inversion locus and the permanently heterozygous locus. Mutations are at mutation-selection equilibrium frequencies. Inversions of 2 Mb are introduced at different frequencies in the population, and with different levels of association with 1 of the 2 permanently heterozygous alleles, which therefore generates various initial linkage disequilibrium values (D). Inversions appear more or less linked to a locus with 2 permanently heterozygous alleles; completely linked inversions can therefore only increase up to a maximum frequency of 50%. Linkage strength is indicated by line colors, representing the distance in cM between inversions and the permanently heterozygous alleles/locus. Inversions at more than 50 cM from the permanently heterozygous locus behave like inversions on autosomes. The figure illustrates the case of inversions carrying a number of mutations 20% lower than the population average (*m* = ⌊0.8×*nq*⌋), as frequently observed (S1–S3 Figs). A dominance coefficient of *h* = 0.01 was used for these deterministic simulations. (**A**) Inversion change in frequency. Similar to Figs 2c and S5 but considering inversions in linkage with a locus with 2 permanently heterozygous alleles, and various initial levels of linkage disequilibrium between the inversion locus and the permanently heterozygous locus. (**B**) Change in the level of linkage disequilibrium (*D*) between the inversion locus and the permanently heterozygous locus. If there is no initial linkage disequilibrium (i.e., inversions are introduced at the same frequency in linkage with each of the 2 permanently heterozygous alleles), the inversion does not spread. As soon as there is an initial linkage disequilibrium, even very small, this linkage disequilibrium increases and the inversion spreads. Here, the initial linkage disequilibrium is artificially generated by introducing the inversions with different levels of association with a permanently heterozygous allele. In finite populations, this non-null initial linkage disequilibrium can easily be generated by founder-like effects (an inversion typically appearing on a single haplotype) or by the random fluctuations of inversion frequency induced by drift. See S1 Appendix, section 6, for modeling details. The script used to produce this figure is available on GitHub.
(PNG)

S7 Fig Deterministic trajectory of inversion frequency when in linkage to a permanently heterozygous locus with 3 alleles. Similar to Figs 2c and S3–S5 but considering inversions in linkage to a locus with 3 permanently heterozygous alleles. Trajectory of inversions depending on the selection and dominance coefficients of their mutations and their degree of linkage to the permanently heterozygous locus. Mutation frequencies are at mutation-selection equilibrium (see Methods) with a mutation rate of *μ* = 10^−8^. Inversions of 2 Mb are introduced at a 0.01 frequency in linkage with 1 of the 3 permanently heterozygous alleles. The figure illustrates the case of inversions carrying a number of mutations 20% lower than the population average (*m* = ⌊0.8×*nq*⌋), as frequently observed in simulations (S1–S3 Figs). Linkage strength is indicated by line colors, representing the distance in cM between inversions and permanently heterozygous alleles. When fully linked to the permanently heterozygous locus (0 cM), inversions can increase up to a maximal frequency of 1/3, meaning that they are fully associated to 1 of the 3 permanently heterozygous alleles. See S1 Appendix, section 7, for modeling details. The script used to produce this figure is available on GitHub.
(PDF)

S8 Fig Deterministic trajectory of inversion frequency when in linkage with an overdominant locus with no permanently heterozygous alleles. Similar to Fig 2C but with an overdominant locus with 2 alleles. Trajectory of inversions depending on the selection and dominance coefficients of their mutations and the strength of selection acting on the overdominant locus (with no permanently heterozygous alleles). Mutation frequencies are at mutation-selection equilibrium (see Methods) with a mutation rate of *μ* = 10^−8^. The figure illustrates the case of 2-Mb inversions carrying a number of mutations 20% lower than the population average (*m* = ⌊0.8×*nq*⌋). Inversions appear in full linkage (*r* = 0) with 1 of the 2 alleles at an overdominant locus where both homozygotes have reduced fitness (1−*s*_2_; when *s*_2_ is close to 1, homozygotes suffer from a strong reduction in fitness and are therefore rare). See S1 Appendix, section 5, for modeling details. The script used to produce this figure is available on GitHub.
(PDF)

S9 Fig Expected equilibrium frequency of 2-Mb inversions as a function of selection and dominance coefficients. Expected equilibrium frequency of all 2-Mb inversions that can occur capturing the male-determining allele in an XY system (right column) or on an autosome (left column). Therefore, this is similar to Fig 2D but considering all inversions, i.e., inversions less loaded and more loaded than average. The expected equilibrium frequency was calculated using Eqs 4 and 5 (Methods). The frequency displayed for Y-linked inversions is the frequency of inversions in the population of Y chromosomes. Y-linked inversions become fixed (equilibrium frequency = 1) when *m*<*nq* and are lost (equilibrium frequency = 0) when *m*>*nq* (see Methods and main text). These 2 events have nearly equal probabilities when *nq* is high (Figs 2B and S1), and therefore the expected equilibrium frequency of Y-linked inversion is often around 0.5. The script used to produce this figure is available on GitHub.
(PDF)

S10 Fig Evolution of 2-Mb inversions in stochastic simulations during 10,000 generations. Similar to Fig 3A but with other parameter values (*s*, *h*). For each parameter combination, 10,000 inversions of 2,000 kb were simulated in a population harboring an XY locus (2 alleles, one being permanently heterozygous). Populations of 1,000 individuals were simulated. We considered inversions fully linked to the Y sex-determining allele, fully linked to the X sex-determining allele or on an autosome. Only inversions not lost after 20 generations are displayed. In contrast to Fig 3A, the overall frequency of Y-linked and X-linked inversion is displayed (instead of the frequency of inversion in the Y chromosome population). Inversions fixed on the Y chromosome have therefore a 0.25 frequency (and 0.75 for X-linked inversions). For each parameter combination, the number of inversions lost and segregating or fixed at the end of the simulation is indicated above lines (« c =. . . »). Because *N* = 1,000, mutations with *s* = 0.001 (i.e., 1/N) are nearly neutral, which explains that X-linked or autosomal inversions can spread in the population, in contrast to what is observed with *s* > 0.001. The dataset and script used to produce this figure are available on Figshare (doi: 10.6084/m9.figshare.19961033) and GitHub.
(PDF)

S11 Fig Evolution of 2-Mb inversions in stochastic simulations over 10,000 generations in populations of *N* = 10,000 individuals with *s* = 0.01. Similar to Fig 3A and 3B but with *N* = 10,000. (**a**) Change in inversion frequency in stochastic simulations with 10,000 individuals experiencing recessive deleterious mutations at a rate *μ* = 10^−8^, including following inversion occurrence, all mutations having the same dominance and selection coefficients (here, *h* = 0.1 and *s* = 0.01). The figure displays the frequency of inversions on an autosome and on a proto-Y chromosome, each line representing a specific inversion. (**b**) Fluctuations in the mean number of mutations carried by the inverted segments in each of the 10,000 simulations, each line representing 1 simulation. In contrast to what happens with *N* = 1,000 (Fig 3A and 3B), some inversions rise in frequency on the Y chromosome; however, the high population size renders the time for inversion fixation too long, they accumulate deleterious mutations before they can fix and therefore all inversions were lost at the simulation end. The dataset and script used to produce this figure are available on Figshare (doi: 10.6084/m9.figshare.19961033) and GitHub.
(PDF)

S12 Fig Evolution of 2-Mb inversions in stochastic simulations over 10,000 generations in populations of *N* = 10,000 individuals with *s* = 0.001. Similar to S11 Fig but with *s* = 0.001. (**a**) Change in inversion frequency in stochastic simulations with 10,000 individuals experiencing recessive deleterious mutations at a rate *μ* = 10^−8^, including after inversion occurrence, all mutations having the same dominance and selection coefficients (here, *h* = 0.1 and *s* = 0.001). The figure displays the frequency of 10,000 inversions on an autosome and on a proto-Y chromosome, each line representing a specific inversion. (**b**) Fluctuations in the mean number of mutations carried by the inverted segments in each of the 10,000 simulations, each line representing 1 simulation. In contrast to the S11 Fig, several inversions fix on the Y chromosome before they accumulate too many mutations. Inversions take more time to fix than when *N* = 1,000 (Figs 3 and S10). The dataset and script used to produce this figure are available on Figshare (doi: 10.6084/m9.figshare.19961033) and GitHub.
(PDF)

S13 Fig The accumulation of mutations in autosomal and sex-linked inversions in finite populations strongly departs from infinite population approximation predictions. (**a–b**) Change in inversion frequency in stochastic simulations with *N* = 1,000 individuals experiencing recessive deleterious mutations at a rate *μ* = 10^−8^ or = 10^−9^, all mutations having the same dominance and selection coefficients (here, *h* = 0.1 and *s* = 0.01). The figure displays the frequency of 2-Mb inversions on an autosome and on a proto-Y chromosome. Each line represents the trajectory of one of these 10,000 simulations under each set of parameters. The lines end when no more inverted segments segregate in the population (i.e., when all inversions are lost or fixed). For *μ* = 10^−8^, the same plots as in Fig 3A are presented but with a different scale for autosomal inversions. (**c–d**) Minimum number of mutations found in inverted segments in stochastic simulations. Note the different scales of the x axes in panels c and d: as shown in panel a–b, no inversion segregated until the end of the simulation in the autosome (10,000 generations), thereby explaining the reduced x axis. (**e–f**) Same as panel c–d but displaying the mean number of mutations in inverted segments (instead of the minimum number). For *μ* = 10^−8^, the same plots as in Fig 3B are presented (but with different scales for autosomal inversions). (**g**) Deterministic change in inversion mutation number in infinite populations for a mutation rate of *μ* = 10^−8^ or *μ* = 10^−9^, as defined by Nei and colleagues (1967), and by Connallon and Olito (2021). All mutations were considered to have the same dominance and selection coefficients (here, *h* = 0.1 and *s* = 0.01). We considered here that inverted segments were initially mutation free. This shows that the observed accumulation of mutations in inversions on autosomes or on the Y chromosome strongly departs from the infinite population expectations.
(PDF)

S14 Fig Evolution of 2-Mb recombination suppressors in linkage with a locus with 2 permanently heterozygous alleles in stochastic simulations during 10,000 generations. Similar to Fig 3A but with a locus with 2 permanently heterozygous alleles (instead of one in the case of the XY system) and with other recombination suppressors than chromosomal inversions. For each parameter combination, 10,000 recombination suppressors of 2 Mb were simulated. These recombination modifiers suppress recombination within the segment in which they reside, both when heterozygous and when homozygous. These recombination suppressors were either fully linked (*r* = 0) or fully unlinked (*r* = 0.5) to a locus with 2 permanently heterozygous alleles; recombination suppressors fully linked to 1 of the 2 permanently heterozygous alleles can spread to a maximum frequency of 50%. Only recombination suppressors not lost after 20 generations were considered for this figure. At the end of the simulation, all recombination suppressors display either a 0.0 or a 0.5 frequency, meaning they are either lost or fixed to a given permanently heterozygous allele. The number of recombination suppressors in each state at the end of the simulation is indicated above lines (« c =. . . »). Populations of *N* = 1,000 individuals were simulated. The dataset and script used to produce this figure are available on Figshare (doi: 10.6084/m9.figshare.19961033) and GitHub.
(PDF)

S15 Fig Proportions of inversions in stochastic simulations that were fixed after 10,000 generations for different parameter value combinations and with *N* = 1,000. Similar to Fig 3 but considering different sizes of inversions. The dataset and script used to produce this figure are available on Figshare (doi: 10.6084/m9.figshare.19961033) and GitHub.
(PDF)

S16 Fig Proportions of inversions in stochastic simulations that were fixed after 10,000 generations for different parameter value combinations with *N* = 10,000. Similar to Figs 3 and S15 but with *N* = 10,000 and for different sizes of inversions. The dataset and script used to produce this figure are available on Figshare (doi: 10.6084/m9.figshare.19961033) and GitHub.
(PDF)

S17 Fig Proportions of inversions in stochastic simulations that were fixed after 10,000 generations for different parameter value combinations with *N* = 1,000. Similar to Figs 3 and S15 but considering that mutations segregating in the genome have their fitness effects drawn from a gamma distribution with a shape of 0.2, and their dominance coefficient *h* randomly sampled among 0, 0.001, 0.01, 0.1, 0.25, 0.5 with uniform probabilities. Simulations were run considering that the mean of the selection coefficient values (mean of the gamma distribution) was either 0.001, 0.01, 0.1, or 0.5. The dataset and script used to produce this figure are available on Figshare (doi: 10.6084/m9.figshare.19961033) and GitHub.
(PDF)

S18 Fig Evolution of fusion-mimicking mutations in stochastic simulations during 10,000 generations. (**a**) Graphical representation of the chromosome fusions simulated. The fusion-mimicking mutations result in the linkage of 2 chromosomes of each pair and in the suppression of recombination in heterozygotes over 1 Mb in the fused side of each chromosome. Therefore, these mutations behave as 2-Mb inversions that would also lead to chromosome fusion. (**b**) Similar to Fig 3A but considering the fusion-mimicking mutations instead of inversions. Simulations where performed with *N* = 1,000, *μ* = 5×10^−8^, and *s* = −0.01. For each parameter combination, 10,000 fusion-mimicking mutations were simulated in a population harboring a pair of autosomes and a pair of XY-like nonrecombining sex chromosomes (females being XX and males XY) with a 1-Mb recombining region on each sex-chromosome side (mimicking pseudoautosomal regions). Only fusions not lost after 20 generations are displayed. The displayed frequency of the fused chromosomes is their frequency among the chromosomes of the same type, e.g., a Y-autosome fusion at 1.0 frequency means that all Y chromosomes are fused with an autosome. The dataset and script used to produce this figure are available on Figshare (doi: 10.6084/m9.figshare.19961033) and GitHub.
(PDF)

S19 Fig Fraction of Y-linked inversions spreading or fixed after 10,000 generations depending on the mean number of mutations segregating in the region where they appear. For each parameter combination, 10,000 inversions fully linked to a Y sex-determining allele (permanently heterozygous) were simulated. The number of mutations displayed here represents the mean number of mutations in haplotypes of the whole population in the region covered by inversions and not the number of mutations in the inversions themselves. Inversions have higher chances of spreading when they appear in mutation-dense regions. Populations of 1,000 individuals were simulated. The X axis is log-scaled. The dataset and script used to produce this figure are available on Figshare (doi: 10.6084/m9.figshare.19961033) and GitHub.
(PDF)

S20 FigFraction of 1-Mb less-loaded inversions that went to fixation depending on the heterozygous fitness cost they are associated with.The heterozygous fitness cost is defined in such a way that $W_{NI}^{\eta }=W_{NI}(1-\eta )$, with $W_{NI}^{\eta }$ the fitness of individual heterozygotes for the inversion with the cost (see S1 Appendix, section 10). Simulations were performed with *N* = 1,000, *μ* = 5×10^−9^, and *s* = −0.01. A Y-linked inversion was considered fixed if it was present on all Y chromosomes. Y-linked inversions become fixed (equilibrium frequency = 1) when *m*<*nq*−ln(1−*η*)/(−*hs*) and are lost (equilibrium frequency = 0) when $m>nq-\frac{\ln\left(1-\eta \right)}{-hs}$. Autosomal inversions become fixed (equilibrium frequency = 1) when *m*<*nqh*/(1−*h*)+ln(1−*η*)/*s*(*h*−1) and are lost (equilibrium frequency = 0) when *m*>*nq*−ln(1−*η*)/(−*hs*) (see S1 Appendix, section 10). Parameters resulting in *nq* = 1,2,3,…,6 expected mutations are highlighted by red lines (top line, *nq* = 1; bottom line, *nq* = 6). The script used to produce this figure is available on GitHub.(PDF)

S21 FigFraction of 5 Mb less-loaded inversions that went to fixation depending on the heterozygous fitness cost they are associated with.The heterozygous fitness cost is defined in such a way that $W_{NI}^{\eta }=W_{NI}(1-\eta )$, with $W_{NI}^{\eta }$ the fitness of individual heterozygotes for the inversion with the cost (see S1 Appendix, section 10). Simulations were performed with *N* = 1,000, *μ* = 5×10^−9^, and *s* = −0.01. A Y-linked inversion was considered fixed if it was present on all Y chromosomes. Y-linked inversions become fixed (equilibrium frequency = 1) when *m*<*nq*−ln(1−*η*)/(−*hs*) and are lost (equilibrium frequency = 0) when $m>nq-\frac{\ln\left(1-\eta \right)}{-hs}$. Autosomal inversions become fixed (equilibrium frequency = 1) when *m*<*nqh*/(1−*h*)+ln(1−*η*)/*s*(*h*−1) and are lost (equilibrium frequency = 0) when *m*>*nq*−ln(1−*η*)/(−*hs*) (see S1 Appendix, section 10). Parameters resulting in *nq* = 3, 4, 5, or 6 expected mutations are highlighted by red lines (top line, *nq* = 3; bottom line, *nq* = 6). The script used to produce this figure is available on GitHub.(PDF)

S22 Fig Proportions of inversions in stochastic simulations that were fixed after 10,000 generations for different parameter value combinations with *N* = 1,000 and in populations with haplodiplontic life cycles. Similar to Fig 3C but considering species with different life cycles. Four life cycles were considered: fully diploid (as used throughout this study) and haplodiplontic with occurrence of a haploid phase every x generation, with x being 2, 3, or 10. Simulations were performed with *N* = 1,000, *μ* = 5×10^−9^, and *s* = −0.01. This shows that inversions are less likely to spread and fix in species with extended haploid phases, as such life cycles lead to more efficient purge of deleterious recessive mutations. See S23 Fig for the variation in mutation load in populations with different life cycles. The dataset and script used to produce this figure are available on Figshare (doi: 10.6084/m9.figshare.19961033) and GitHub.
(PDF)

S23 Fig Mutation load evolution in populations with different life cycles during the burn-in phase. For the simulations of the effect of different life cycle on the fate of inversions (S22 Fig), for each set of parameter values, one simulation was run and used as the initial state after a burn-in period of 15,000 generations (see Methods). We display here the evolution of the mutation load during the burn-in phase for populations with different life cycles. Four haplodiplontic life cycles were considered, with a haploid phase every x generation, with x being 2, 3, 10, or 100. Each trajectory represents 1 simulation. (**a**) Total number of mutations segregating across the genome in the population. (**b**) Mean number of segregating mutations in the genome in diploid individuals. (**c**) Mean frequency of mutations in the population. This shows that populations with an extended or frequent haploid phase tend to have a reduced mutation load compared to populations with rare or brief haploid phases. The dataset and script used to produce this figure are available on Figshare (doi: 10.6084/m9.figshare.19961033) and GitHub.
(PDF)

S24 Fig Successive accumulation of inversions around a male-determining allele in an XY system, leading to the formation of nonrecombining sex chromosomes. Similar to Fig 4 but displaying the result of another simulation and with a population of *N* = 10,000 individuals. A simulation of *N* = 10,000 individuals, each with 2 pairs of 100-Mb chromosomes, during 100,000 generations. Chromosome 1 harbors an X/Y sex-determining locus at 50 Mb (individuals are XX or XY). Each generation, 1 inversion appears on average in the whole population, in an individual sampled uniformly at random, with the 2 recombination breakpoints sampled uniformly at random among *k* = 100 potential breakpoints. (**a**) Overview of chromosomal inversion frequency and position for 10 different generations. Square width represents inversion position and square height inversion frequency. Inversions appearing on the Y chromosome are depicted in yellow, those appearing on the X chromosomes in gray. The colors are not entirely opaque, so that regions with overlapping inversions appear darker. Loss of previously fixed inversions are due to beneficial reversion occurrence and selection. (**b**) Changes in the relative rate of recombination over the entire course of the simulation. The numbers of recombination events occurring at each position (binned in 1-Mb windows) are recorded at the formation of each offspring, across all homologous chromosomes in the population. To illustrate the evolution of recombination suppression between the sex chromosomes, only recombination events between the X and the Y chromosomes are shown for chromosome 1 (i.e., not the recombination events between the 2 X chromosomes in females). Unlike chromosome 1, chromosome 2 harbors no permanently heterozygous allele. All inversions on this chromosome suffer from homozygosity disadvantage and very few inversions therefore become fixed on chromosome 2. The dataset and script used to produce this figure are available on Figshare (doi: 10.6084/m9.figshare.19961033) and GitHub.
(PDF)

S25 Fig Population evolution during the burn-in phase. For the simulations of the effect of different parameters (notably *h* and *s*) on the fate of inversions (Figs 3 and S10–S13, notably), for each set of parameter values, 1 simulation was run and used as the initial state after a burn-in period of 15,000 generations (see Methods). We display here the evolution of the population during the burn-in phase. Each trajectory represents the state of one simulation. (**a**) Number of mutations segregating in the genome. (**b**) Mean frequency of segregating mutations in the genome. This shows that each population had reached an equilibrium state at the end of the burn-in period. The dataset and script used to produce this figure are available on Figshare (doi: 10.6084/m9.figshare.19961033) and GitHub.
(PDF)

S1 Appendix Supplementary methods. (PDF)
